# Deep Learning-Based Magnetic Resonance Imaging in Diagnosis and Treatment of Intracranial Aneurysm

**DOI:** 10.1155/2022/1683475

**Published:** 2022-06-13

**Authors:** Xiubing Lei, Yang Yang

**Affiliations:** ^1^Medical College of Panzhihua University, Panzhihua, 617000 Sichuan, China; ^2^Clinical Medical College of Panzhihua University, Panzhihua, 617000 Sichuan, China

## Abstract

This study was focused on the positioning of the intracranial aneurysm in the magnetic resonance imaging (MRI) images using the deep learning-based U-Net model, to realize the computer-aided diagnosis of the intracranial aneurysm. First, a network was established based on the three-dimensional (3D) U-Net model, and the collected image data were input into the network to realize the automatic location and segmentation of the aneurysm. The 3D convolutional neural network (CNN) network can extract the aneurysm blood vessels to locate and identify the areas of possible aneurysms. Next, 40 patients highly suspected of intracranial aneurysm were selected as research subjects, and they were subjected to magnetic resonance angiography (MRA) and digital subtraction angiography (DSA) examinations. The results showed that based on the U-Net algorithm model, 40 patients' hemangiomas were completely contained in the labeling bounding box, one patient's hemangioma was at the edge of the labeling bounding box, and 4 patients' hemangiomas were outside the labeling box. The final accuracy coefficient was 88.9%, and it was in good agreement with the doctor's manual labelling results. Under the 3D CNN network test, the sensitivity, specificity, and accuracy of DSA for intracranial aneurysm were 91.46%, 86.01%, and 90.2%, respectively; the sensitivity, specificity, and accuracy of MRA for intracranial aneurysm were 95.87%, 100%, and 97.19%, respectively. In conclusion, the 3D CNN can successfully realize the positioning of intracranial aneurysm in MRA images, providing a certain theoretical basis for subsequent imaging diagnosis of aneurysm.

## 1. Introduction

With the development of society and the improvement of people's living standards, cerebrovascular diseases have gradually become a high-risk disease. Intracranial aneurysm is representative of cerebrovascular diseases. Its incidence of ranks third among cerebrovascular diseases, second only to cerebral thrombosis and high-pressure cerebral hemorrhage [1, 2]. Relevant data show that for every 100 adults in China, 7 are aneurysm carriers. Intracranial aneurysm refers to the tumor-like protrusions formed by weak blood vessels in the local cerebral arteries. It is common in people between 30 and 60 years old. Clinically, intracranial aneurysm is the main cause of subarachnoid hemorrhage (SAH), and 70% patients of intracranial aneurysm suffer from SAH [3, 4]. Intracranial aneurysm is usually found in the arteries at the base of the brain, and the location here is generally called the ring of the arteries at the base of the brain, also known as the Willis ring. It involves anterior communicating artery, bilateral anterior cerebral artery beginning segment, bilateral internal carotid artery end segment, bilateral posterior communicating artery, and bilateral posterior cerebral artery beginning segment [5–7]. 80% of the aneurysms occur in the posterior Willis ring.

At present, the commonly used methods to examine aneurysms include digital subtraction angiography (DSA), magnetic resonance angiography (MRA), and other imaging methods [8, 9]. These cerebral angiography methods are mainly based on visual observation. CT angiography can confirm the existence of aneurysm, and it is safe and fast. Additionally, it is painless, does not affect intracranial pressure, and can be performed repeatedly. However, it is not as good as cerebral angiography in identifying the size or location of the aneurysm [10, 11]. DSA only retains the vascular images, which can realize the positioning of vascular lesions and has huge advantages in judging the direction of blood flow [12, 13]. MRA uses electromagnetic waves to generate a two-dimensional or three-dimensional structure image. It is a kind of tomography and uses magnetic resonance phenomenon to obtain electromagnetic signals from the human body and reconstruct human body information. In clinical practice, MRA is nonradiative, noninvasive, and comprehensive [14], while MRA depends on the subjective judgment of radiologists in the examination of cerebral aneurysms, and the sensitivity of the radiologist's clinical judgment is about 70% [15], because fatigue and subjective judgment will affect the results of the examination, leading to the occurrence of missed diagnosis and misdiagnosis. Therefore, the realization of computer-aided diagnosis is extremely important for the diagnosis and treatment of intracranial hemangioma.

With the rapid development of convolutional neural networks, superresolution reconstruction algorithms based on deep learning have achieved very good results in the field of natural images, and these methods have also been extended to the field of medical images by researchers in recent years. The computer-aided diagnosis of MRA mainly relies on the convolutional neural network (CNN) in the deep learning. Different from the superresolution reconstruction of natural images, 3D CNN is mostly used for superresolution reconstruction of 3D medical images. Both the U-Net model and the 3D CNN network use full convolutional networks for image detection. The introduction of deep learning in the labeling process can improve the detection and diagnosis effect of cerebral hemangioma [16–18]. CNN can be divided into 2D convolution and 3D convolution according to the dimension of the convolution kernel. Usually, 2D convolution is used on data with two-dimensional structure such as natural images, while 3D convolution is often used in video and medical images with 3D properties.

Above, in this study, a deep learning-based network algorithm model was established first to detect intracranial aneurysm, and the two inspection methods of MRA and DSA were compared for the diagnosis accuracy of intracranial aneurysm. The primary objective of the study was to analyze the application value of MRA in the clinical diagnosis of intracranial aneurysm, expected to provide a theoretical basis for clinical diagnosis and treatment of cerebral aneurysm.

## 2. Materials and Methods

### 2.1. Research Subjects

Forty patients who were highly suspected of intracranial aneurysm were selected as research subjects, including 24 female patients and 16 male patients, ranging in age from 24 to 77 years old, with an average age of 53.1 years old. They were all subjected to the MRA examination and then the DSA imaging examination and data were collected after the examination. This study had been approved by ethics committee of hospital, and the patients and their families signed the informed consents.

Inclusion criteria: (1) patients with typical symptoms of intracranial aneurysm [19] but not diagnosed with intracranial aneurysm; (2) there were no other tumors, cysts, or tuberculomas in the brain. Exclusion criteria: (1) patients who were diagnosed with intracranial aneurysm and those who were determined not to have intracranial aneurysm; (2) there were other tumors, cysts, and tuberculomas in the brain; (3) metal objects were implanted in the body.

### 2.2. MRA and DSA Inspection Methods and Image Analysis

The MRI scanning equipment adopted 1.5 T MRI scanner with 8-channel head coil. The patient was in a supine posture on the examination table, with the head fixed. During the contrast-enhanced MRA, coronal 3D TRICKS scan was performed, and the scan range was determined according to the direction of the blood vessel. The first step was to perform a three-dimensional fast gradient back mask scan on the patient, then, the scan was paused, and contrast agent was injected. At this time, drug injection and scanning were performed spontaneously, and a total of 14 time phases were scanned. After scanning, the image data of each phase would be automatically subtracted from the mask, and at this time, enhanced blood vessel images of different phases were obtained.

DSA used 2.0 angiography machine, and the Seldinger method was used for puncture [20]. After the blood vessel was successfully punctured, the catheter was inserted, and the angiographic catheter was placed into the vertebrobasilar artery and common carotid artery, respectively, for cerebrovascular angiography. Next, 3D-DSA imaging examination was performed on the internal carotid artery.

The imaging data obtained from MRA and DSA examinations were independently reviewed and checked by two associate senior radiologists and a neurosurgeon. The two imaging examination methods, MRA and DSA, were compared for the sensitivity, specificity, and accuracy diagnosis.

### 2.3. Intracranial Aneurysm Diagnostic Criteria

Positive criteria: (1) the intracranial aneurysm was diagnosed by surgical examinations such as endovascular embolization; (2) the presence of aneurysm must be confirmed in both MRA and DSA tests, and the aneurysm was clearly displayed.

Negative criteria: (1) all examination methods showed no intracranial aneurysm; (2) in both MRA and DSA imaging examinations, the intracranial arteries were clear and complete, and no aneurysms were seen.

### 2.4. Intracranial Aneurysm Positioning Based on U-Net Model

Clinical diagnosis of intracranial aneurysm often requires doctors to observe its MRA images repeatedly. The process takes a lot of time and energy. In this study, a 3D U-Net model algorithm based on deep learning is introduced to quickly diagnose patients suspected of having intracranial aneurysm, and label the area where there may exist intracranial aneurysm. In the 3D U-Net model, the input original data is 3D TOF MRA image sequence, and the output part is the three-dimensional data with the bounding box of the aneurysm, as shown in Figure 1.

As shown in Figure 2, the U-Net network model consists of two paths, namely, a contraction path and an expansion path. U-Net can directly add the features corresponding to the contraction layer to the expansion layer, so that the features of the image will not be lost and merge with the features of the expansion layer to output the segmented image. Because the U-Net network model is sensitive to the initial value, a specification layer is added after each layer of the U-Net network, which reduces the sensitivity of the network to the initial value and speeds up the convergence of the model.

### 2.5. Intracranial Aneurysm Recognition Based on 3D CNN Network

3D CNN is applied to intracranial aneurysm classification, and Figure 3 shows the network structure of the model. Because of the number of samples, the network structure built in this study is relatively simple to avoid overfitting. The structure consists of two three-dimensional convolutional layers, two three-dimensional pooling layers, and a fully connected layer. The number of convolution kernels of the two three-bit convolutional layers are 16 and 32, and the size is 3 × 3 × 3, and the step size is 1, and the size of the two three-dimensional pooling layer filters is 2 × 2 × 2. The length is 1, and the feature dimension of the fully connected layer is 15. The loss function used in the 3D CNN network algorithm is binary cross entropy.

### 2.6. Statistical Processing

SPSS19.0 software was used for statistical analysis. Measurement data conforming to the normal distribution were represented by the mean ± standard deviation, and the difference between groups was analyzed by independent sample *t* test; measurement data that did not conform to the normal distribution were represented by the median value and four-point position, and nonparametric rank sum test was used to analyze the difference between groups. Count data was expressed by *n* (%), and the comparison of differences between groups was analyzed by chi-square test. *P* < 0.05 indicated that the difference was statistically significant.

## 3. Results

### 3.1. Positioning of Intracranial Aneurysm Based on U-Net Model

After the hemangioma that was slender, too large, and too small was excluded, 45 patients' MRA image data were collected, and the image format was BMP. The introduction of the U-Net algorithm model realized the automatic labeling of the suspected hemangioma in the patient's MRA image and GPU acceleration and Adam method were used to train the automatic labeling U-Net algorithm. After comparison with the manual labeling results, it was found that 40 patients' hemangiomas were completely contained in the labeling bounding box, one patient's hemangioma was at the edge of the labeling bounding box, and 4 patients' hemangiomas were outside the labeling box. The final accuracy coefficient was 88.9%, and it was in good agreement with the doctor's manual labelling results.  Figure 4 was the schematic diagram of automatic labeling, and Figure 5 was the manual labeling by doctors.

### 3.2. Recognition Results of Intracranial Aneurysm Based on 3D CNN Network

For the 3D CNN network that has been built, the GPU acceleration was used to train the CNN, with the learning momentum set to 0 and the learning rate set to 0.0000001. The weight of the network was optimized using the Adam method, and all sample images input to the network one time were called an iteration, and the maximum number of iterations was 1000 times.

Direct testing and voting testing were performed on the trained 3D CNN network. The AUC value of the direct testing was 0.9317, as shown in Figure 6, the accuracy of the direct testing was 87.13%, and the sensitivity was 84.57%; after voting classification, the accuracy was 93.13%, and the sensitivity was 93.77%. The sensitivity and accuracy of the test samples were improved to a certain extent after voting (Figure 6).

### 3.3. Diagnosis of Patients with Intracranial Aneurysm

In this study, 29 patients were diagnosed as intracranial aneurysm by surgical intervention, and 5 patients were diagnosed as having intracranial aneurysm under the combined imaging examination of MRA and DSA instead of the surgical intervention, of whom 3 patients fully met the above diagnostic criteria for intracranial aneurysm, and 6 patients were found to have no aneurysms after the combined examination. A total of 34 patients with aneurysms were diagnosed, and 42 aneurysms were clearly detected, which existed in various parts of the cerebral blood vessels. As shown in Figure 7, there were 17 anterior communicating arterial aneurysms (40.4%), 11 posterior communicating aneurysms (26.2%), 5 internal carotid aneurysms (11.9%), 4 anterior cerebral aneurysms (9.5%), 4 middle cerebral aneurysms (9.5%), and 2 vertebrobasilar aneurysms (4.8%).

### 3.4. Comparison of Diagnosis Results between MRA and DSA in Patients with Intracranial Aneurysm

As shown in Figure 8, in the DSA examination of 40 patients, a total of 30 positive patients were detected, of which 2 were false positives, and 3 were false negatives after subsequent confirmation. The sensitivity, specificity, and accuracy of DSA for intracranial aneurysm were 91.46%, 86.01%, and 90.2%, respectively.

In the MRA examination of 40 patients, 33 positive patients were detected, of which 1 case was false positive, and 7 cases were false negatives after subsequent confirmation. The sensitivity, specificity, and accuracy of MRA for intracranial aneurysm were 95.87. %, 100%, and 97.19%, respectively (Figure 9).

In MRA examination, 5 cases of intracranial aneurysm with hemorrhage were not found, while the lesions of these 5 patients were diagnosed normally in the DSA examination; there were 6 cases of intracranial aneurysm correctly diagnosed by MRA, but DSA only correctly diagnosed 2 cases of intra-aneurysm hemorrhage (Figure 10).

## 4. Discussion

The disability rate of patients with aneurysm rupture for the first time after suffering from intracranial aneurysm is very high, and some patients die of rebleeding from the aneurysm. Early surgical treatment can effectively avoid the bleeding of aneurysm, so early clinical diagnosis of intracranial aneurysm is of vital importance to improve and reduce the mortality of intracranial aneurysm. DSA, as the gold standard for the diagnosis of intracranial aneurysm, has the characteristics of high accuracy, but its shortcomings are also obvious. Its inspection time is long, and it is traumatic and costly. As a result, it cannot be accepted by all patients [21]. With the gradual development of medical imaging technology, MRA has been gradually improved and applied as a noninvasive diagnostic method for intracranial aneurysm. MRA can clearly display the structure of cerebral blood vessels and has important clinical value for the diagnosis of intracranial aneurysm. In recent years, it has been increasingly used [22].

With the dual development of deep learning technology and medical imaging technology, deep learning is frequently used in the field of medical image analysis, and CNNs can effectively identify lesions and has huge advantages in the identification and labeling of special lesions [23]. In this study, after comparison with the manual labeling results, it was found that 40 patients had hemangiomas that were completely contained within the labelled bounding box, 1 patient had hemangiomas at the edge of the labelled bounding box, and 4 patients had hemangiomas outside the labelled box. The final accuracy coefficient was 88.9%, which was in good agreement with the doctor's manual labeling results. In the 3D CNN network test, the sensitivity, specificity, and accuracy of DSA for intracranial aneurysms were 91.46%, 86.01%, and 90.2%, respectively; while those of MRA were 95.87%, 100%, and 97.19%, respectively. Therefore, the CNN is far more sensitive to intracranial aneurysm than the manual examination.

MRA can clearly display the cerebral vascular structure mainly by the flow effect of blood and the contrast of static tissue, and its principle is mainly the phase change and flow enhancement effect [24]. The results of this study showed that the diagnostic sensitivity, specificity, and accuracy of MRA were significantly higher than DSA, so the clinical application of MRA for intracranial aneurysm diagnosis has high value.

## 5. Conclusion

The study was to use deep learning to automatically label intracranial aneurysm MRA images and to further evaluate its value in the diagnosis of intracranial aneurysm. The results showed that the 3D CNN network can realize the location and recognition of aneurysms. The results show that based on the U-Net algorithm model is in good agreement with the doctor's manual labelling results. Its diagnostic sensitivity, specificity, and accuracy are better than DSA. In conclusion, the 3D CNN can successfully realize the positioning of intracranial aneurysm in MRA images, providing a certain theoretical basis for subsequent imaging diagnosis of aneurysm. However, some limitations in the study should be noted. The sample size is small, which will reduce the power of the study. In the follow-up, an expanded sample size is necessary to strengthen the findings of the study.

## Figures and Tables

**Figure 1:** Schematic diagram of neural network input and output.

**Figure 2:** U-Net network structure diagram.

**Figure 3:** 3D CNN neural network structure diagram.

**Figure 4:** U-Net algorithm model automatic labeling diagram. (a) Unlabeled; (b) the suspected aneurysm area automatically labelled by the algorithm.

**Figure 5:** Comparison between automatic and manual labeling results. Unlabeled (a), manual labeling by the doctor (b), and automatic labeling by the algorithm (c).

**Figure 6:** Accuracy (ACC) and sensitivity (SEN) of 3D CNN network.

**Figure 7:** Distribution of hemangiomas.

**Figure 8:** Comparison of DSA and the gold standard.

**Figure 9:** Comparison of MRA and the gold standard.

**Figure 10:** Comparison of diagnosis results between MRA and DSA in patients with intracranial aneurysm.

## Data Availability

The data used to support the findings of this study are available from the corresponding author upon request.
